# Application of U-Net with Global Convolution Network Module in Computer-Aided Tongue Diagnosis

**DOI:** 10.1155/2021/5853128

**Published:** 2021-11-18

**Authors:** Meng-Yi Li, Ding-Ju Zhu, Wen Xu, Yu-Jie Lin, Kai-Leung Yung, Andrew W. H. Ip

**Affiliations:** ^1^School of Computer Science, South China Normal University, Guangzhou, Guangdong 510631, China; ^2^School of Geography, South China Normal University, Guangzhou, Guangdong 510631, China; ^3^General ICU of Lingnan Hospital, The Third Affiliated Hospital of Sun Yat Sen University, Guangzhou, Guangdong 510631, China; ^4^Department of Traditional Chinese Medicine, Sun Yat Sen Memorial Hospital, Sun Yat Sen University, Guangzhou, Guangdong 510631, China; ^5^Department of Industrial and Systems Engineering, Hong Kong Polytechnic University, Hong Kong 999077, China; ^6^Department of Mechanical Engineering, University of Saskatchewan, Saskatoon, Canada M4Y1M7

## Abstract

The rapid development of intelligent manufacturing provides strong support for the intelligent medical service ecosystem. Researchers are committed to building Wise Information Technology of 120 (WIT 120) for residents and medical personnel with the concept of simple smart medical care and through core technologies such as Internet of Things, Big Data Analytics, Artificial Intelligence, and microservice framework, to improve patient safety, medical quality, clinical efficiency, and operational benefits. Among them, how to use computers and deep learning technology to assist in the diagnosis of tongue images and realize intelligent tongue diagnosis has become a major trend. Tongue crack is an important feature of tongue states. Not only does change of tongue crack states reflect objectively and accurately changed circumstances of some typical diseases and TCM syndrome but also semantic segmentation of fissured tongue can combine the other features of tongue states to further improve tongue diagnosis systems' identification accuracy. Although computer tongue diagnosis technology has made great progress, there are few studies on the fissured tongue, and most of them focus on the analysis of tongue coating and body. In this paper, we do systematic and in-depth researches and propose an improved U-Net network for image semantic segmentation of fissured tongue. By introducing the Global Convolution Network module into the encoder part of U-Net, it solves the problem that the encoder part is relatively simple and cannot extract relatively abstract high-level semantic features. Finally, the method is verified by experiments. The improved U-Net network has a better segmentation effect and higher segmentation accuracy for fissured tongue image dataset. It can be used to design a computer-aided tongue diagnosis system.

## 1. Introduction

Nowadays, with the rapid development of mobile and wireless networking technologies, the Internet of Things (IoT) has contributed to Wise Information Technology of 120 (WIT 120). Researchers combine modern computer technology with modern medicine and traditional Chinese medicine theory to achieve computer-assisted diagnosis [1–3]. Machine learning and deep learning are also widely used in the medical field. Deep learning, a branch of machine learning, emphasizes the use of multiple levels of abstraction of data [4]. Deep learning is not a new technology; its concept originates from artificial neural networks. In essence, it refers to a kind of effective training method for neural networks with deep structure. Deep learning combines low-level features to form more abstract high-level representation attribute categories or features, to find the distributed feature representation of data. The motivation of studying deep learning is to establish a neural network that simulates the human brain for analytical learning. It simulates the mechanism of the human brain to interpret data, such as images, sounds, and texts. It can automatically abstract and extract low-, mid-, and high-level features directly from the original tongue images to combine from end-to-end [5]. Combining traditional Chinese medicine theory with deep learning technology and analyzing tongue images by constructing a neural network model not only provide a new idea for computer-aided tongue diagnosis but also improve the modernization and automation level of disease diagnosis.

The convolutional neural network plays an important role in the development of deep learning. It plays an irreplaceable role in improving the research level and practical performance of computer vision. In 2012, a historic breakthrough was made in the development of convolutional neural networks. Krizhevsky et al. [6] proposed the famous model named AlexNet by using the Rectified Linear Unit (ReLU) as the activation function. It was the pioneering deep CNN that won the ILSVRC-2012 with a TOP-5 test accuracy of 84.6% and attained a new state-of-the-art performance. At present, a convolutional neural network has replaced the support vector machines (SVMs) of traditional machine learning and has become the most excellent and widely used deep neural network learning model in the field of computer vision, such as image classification, object detection, target tracking, and image segmentation.

Image segmentation can be understood as a method of outputting the category to which each pixel belongs. In object recognition, the number of input layer units is equal to the size of the sample image, and the number of output layer units is equal to the number of categories. During image segmentation, the number of input layer units is the same as object recognition, which is equal to the size of the sample image. But the number of output layer units is equal to the product of the sample image size and the number of categories. The output result of segmentation is the probability that each pixel belongs to each category. Image segmentation objects can be road scenes, face images, and medical images. In 2014, Long et al. [7] designed a fully convolutional network (FCN) that is compatible with images of any size and uses fully supervised learning for image semantic segmentation.

FCN is improved based on VGGNet-16 [8] network. It uses the convolution layer to replace the full connection layer in the traditional CNN and uses the skip layer method to combine the feature map generated by the intermediate convolution layer. Then, the bilinear interpolation algorithm is used to upsampling to convert the rough segmentation results into fine segmentation results. The proposal of FCN provided many scholars with research ideas. Since then, many excellent image segmentation networks have been continuously proposed and widely applied in various fields such as unmanned driving, remote sensing, and medicine.

Tongue diagnosis is one of the distinctive diagnostic methods in traditional Chinese medicine for doctors to understand the physiological functions of the body and cause changes by observing the changes of the tongue and tongue coating of patients. It plays an important role in the clinical diagnosis of traditional Chinese medicine (TCM).

However, the traditional tongue diagnosis is often based on the personal knowledge and experience of doctors, lacking objective evaluation standards. In addition, the valuable experience and tongue image data accumulated in the process of traditional tongue diagnosis cannot be retained scientifically and quantitatively, and the examination results of traditional tongue diagnosis cannot be described scientifically and quantitatively [9], which seriously hinders the application and development of tongue diagnosis. To solve this situation, it is necessary to realize the quantification and standardization of tongue diagnosis. Therefore, TCM tongue diagnosis needs to establish a modern medical system with leading science and technology, objectification, quantification, automation, and exhibition.

At present, more and more medical universities and pharmaceutical enterprises have begun to explore the development route of combining TCM tongue diagnosis with computer science and technology and have achieved a series of scientific research results [10–14]. However, the main research focuses on tongue coating and tongue color, and the research on tongue crack is relatively few.

According to the description in Discrimination of Tongue Image in Traditional Chinese Medicine [15], fissured tongue refers to crisscrossing furrows and cracks on the surface, back of the tongue, or both sides of the tongue, which are called fissured tongue in traditional Chinese medicine. On the one hand, the fissured tongue is caused by Yang deficiency and dampness of the spleen, and on the other hand, it is caused by qi deficiency of the spleen. Because yin deficiency of the spleen and stomach affects the absorption of nutrients in the body, it results in the inability of nutrients to be transmitted to the tongue. Fissured tongue is one of the manifestations of physical malnutrition. The information on tongue crack can not only objectively and accurately reflect the changes of some typical diseases and TCM syndromes but also can be combined with other tongue features to further diagnose diseases. It is very important to study the fissured tongue images.

In this paper, we propose an improved fissured tongue image segmentation model based on the U-Net [16] model. Experiments show that there are some problems in the segmentation of fissured tongue images by the U-Net model. Firstly, in the part of the U-Net encoder, the convolutional neural network with fewer network layers and simpler structure is used. Such a simple network is not very effective in the classification task; it is difficult to extract some abstract high-level features in the image and cannot make full use of the information of the whole image. Therefore, the lack of a coding network makes the final segmentation result not accurate enough. Second, there is less medical image data, the deeper network is difficult to train, and the more complex network is easy to overfitting. Finally, it is easy to lose data during pooling operation, resulting in the unsatisfactory segmentation effect of U-Net.

To solve the above problems, we propose a method based on the combination of U-Net, GCN (Global Convolutional Network) module, and BR (Boundary Refinement) module [17]. During the experiment, the fissured tongue image database is constructed. By comparing different pretraining networks as the encoder and whether to add GCN module and BR module, the comparative experiment is carried out, and the improved U-Net model is proposed. The improved U-Net is tested on the test dataset, and compared with FCN-8s [7], SegNet [18], VGGNet_Unet, and other image segmentation network models, the average intersection union ratio (MIoU) of the improved model is increased by about 15.1%, 30.5%, and 5.3%, respectively.

In summary, the main contribution of this study can be summarized as follows:

1. We have made improvements based on the U-Net network. This method adds GCN and BR modules to the U-Net model. Because large kernels are vital to relieving the contradiction between classification and localization, the improved U-Net structure enables better classification and hence grants the possibility of building a deeper network with higher accuracy.
2. We constructed a database of this study, which was confirmed by consistency assessment by two specialist physicians. We have enhanced the data (eight in the 2D case for the combination of flipping and rotation) to make it available for experiments.
3. We demonstrate the performance of the proposed deep learning architecture by comparing it with the state-of-the-art segmentation methods. Our method outperformed most of the top-ranked methods in terms of segmentation accuracy.

This article is organized as follows. In Section 2, we provide a short review of related work on the topic of typical convolution neural networks and semantic segmentation. In Section 3, we detail the model architecture and the modeling framework.  Section 4 describes the data set we used for training our algorithm. We provide a series of experimental analyses that justifies the design choices for our modeling framework. Last but not least, we present the performance evaluation of our algorithm and comparison with other published results. Finally, Section 5 summarizes the experiment and puts forward the shortcomings of the model and the future development direction.

## 2. Related Work

### 2.1. Common Deep Network Architectures

As we previously stated, a convolutional neural network has made great contributions to the field of image segmentation. It has become a well-known standard to apply convolutional neural networks to segmentation models to realize feature extraction. For that reason, we will focus on these excellent image classification networks in this section.

In 2012, Alex Krizhevsky proposed a very important convolutional neural network model called AlexNet [6]. It won the champion of ILSVRC image classification and attracted wide attention from academia and industry. AlexNet consists of an input layer, five convolution layers, and three full connection layers. Among them, three convolution layers are also maximized.

Inspired by AlexNet, Visual Geometry Group (VGG) is a CNN model introduced by the Visual Geometry Group (VGG) from the University of Oxford. VGGNet [8] explored the relationship between the depth of a convolutional neural network and its performance. By repeatedly stacking 3 × 3 small convolutional kernels and 2 × 2 maximum pooling layer, VGGNet successfully constructed a 16- to 19-layer deep convolutional neural network. Compared to the previous state-of-the-art network structure, VGGNet has significantly reduced the error rate and achieved 2nd place in the ILSVRC 2014 Competition classification project and 1st place in the positioning project. At the same time, VGGNet is very extensible, and migration to other picture data on the generalization is very good.

While VGGNet demonstrated that deepening model structures can help improve network performance, GoogLeNet [19] focused on how to build deeper network structures and introduced a new basic structure, the Inception module (see Figure 1), to increase the width of the network. GoogLeNet V1 is deeper than AlexNet or VGGNet, but its calculation is less than AlexNet and the accuracy is far better than AlexNet, which is a very practical model. The reasons for GoogLeNet V1 to reduce fewer parameters but have a good effect are as follows: one is to remove the final full connection layer and replace it with the global average pooling layer, to make model training faster and reduce overfitting. Moreover, the Inception module improves the utilization of parameters.

As the number of layers increases, deep networks will generally be more difficult to train. When some networks start to converge, they may also have degeneration problems, resulting in saturation of accuracy quickly. The deeper the level, the higher the error rate. Even more surprisingly, the higher error rate caused by this degradation is not overfitting but more layers have been added. In order to solve the degradation problem, a deep residual learning framework was proposed where hundreds of residual networks could be successfully trained. In contrast to a normal neural network, the residual network introduces a cross-layer connection, or shortcut connection, which constructs the residual module (see Figure 2).

ResNet [20] structure can effectively eliminate the increase of error on the training set caused by the layers increase. In addition, the ResNet structure can be well migrated to other network models. GoogLeNet has learned the characteristics of ResNet and proposed Inception V4 and Inception-ResNet-V2 [21]. By integrating these two models, it has achieved excellent results in the ILSVRC dataset. Finally, a series of variant models are generated based on ResNet, such as ResNeXt [22], SEResNet [23], and Feature Pyramid Network (FPN) [24].

### 2.2. Encoder-Decoder

The encoder-decoder networks have been successfully applied to many computers vision tasks, including human pose estimation, object detection, and semantic segmentation [25]. Typically, the encoder-decoder networks consist of two parts: encoder and decoder, in which the encoder gradually reduces the size of the feature map and captures higher-level semantic information, and the decoder gradually recovers the object details and spatial dimensions. The whole structure uses the multiscale features from the encoder module and recovers the spatial resolution from the decoder module.

The U-Net network which is a simple and effective network used in this paper is based on the full convolution network (FCN) network architecture. Its encoder-decoder structure and skip-connection are very classic design methods. The encoder part is responsible for feature extraction, and the decoder part restores the original graphics and gives the prediction of each pixel. Then, the deep information and shallow information are fused by corresponding pixel stitching.

### 2.3. Global Convolutional Network and Boundary Refinement

Semantic segmentation can be considered a per-pixel classification problem. There are two challenges in this task: (1) classification: an object associated with a specific semantic concept should be marked correctly; (2) localization: the classification label for a pixel must be aligned to the appropriate coordinates in the output score map. A well-designed segmentation model should deal with the two issues simultaneously [17].

From the above two aspects, two design principles can be followed: (1) from the point of view of localization, a full convolution structure should be used rather than the full connection layer or global pooling layer; (2) from the point of view of classification, a larger convolution kernel should be used to make the pixel and feature map more closely combined and to enhance the ability to process different transformations. Moreover, too small a convolution kernel will cause a small receptive field. The network cannot cover large targets, which is not conducive to classification.

In order to solve the problem mentioned above, Chao et al. [17] proposed the Global Convolutional Network (GCN) module and Boundary Refinement block (BR) in 2017 (see Figure 3(b)) to replace the postprocessing CRF module. In this paper, the author believes that the network structure should adopt a larger kernel size, so that feature maps and per-pixel classifiers can be closely connected to enhance the ability to cope with transformations. However, a large convolution kernel will lead to a sharp increase in the number of parameters. The paper uses symmetric separated convolution to reduce the model parameters and computation. In this paper, we add the GCN module and BR module on the basis of U-Net. Experimental results show that the addition of this module can effectively improve the segmentation accuracy.

## 3. Methods

As is well known, the diagnosis of the fissured tongue is one of the important diagnostic methods in traditional Chinese medicine. After the recognition of fissured tongue, it is necessary to extract and analyze the characteristics of cracks in the tongue, which can assist doctors to judge the fissured tongue image and to diagnose people's health status through the fissured tongue image in order to achieve more effective treatment and disease prevention.

Because the fissured tongue is an obvious crack groove on the tongue surface, the crack features are usually extracted by setting a threshold for gray and gradient. Wang et al. [26] proposed a fissure extraction method based on Otsu and bot-hat, obtained crack area by the Otsu and extracted fissure by bot-hot, and deleted fake fissures by postprocessing. Yang et al. [27] proposed detection of tongue crack based on distant gradient and prior knowledge. This algorithm uses information of pixel color and gray change fully. Zhang et al. [28] proposed a water flow method suitable for detecting tongue cracks with different widths. This method uses the characteristics of water flow to simulate the flow of water in the terrain to obtain the topographic map, and the tongue crack is detected by calculating the water molecules gathered in the map. It can not only detect the existence of fissures but also quantify the severity from different aspects such as the number of fissures, width, length, and depth.

Furthermore, Chang et al. [29] applied Gradient-Weighted Class Activation Mapping [30] training to test tongue image on ResNet50 network structure to detect and locate cracks. However, some cracks on the face or other parts are also located at the same time; it is needed to improve the accuracy of localization in the future. Liu et al. [31] constructed the model by the fine-tuning method in Faster-RNN deep learning technology and transfer learning technology and evaluated the model effect by using accuracy rate, accuracy rate, and recall rate. The results of image recognition show that the model is not affected by the location of pathological changes in tongue image and has strong adaptability to local feature extraction of tongue image.

Up to now, there is a litter of literature that introduces the extraction and analysis of some features of the fissured tongue [32, 33], but it is far from being systematic and in-depth. Compared with the previous methods, this paper proposes a U-Net [16] network with GCN [17] module to extract cracks features and identify cracks features on the tongue from the perspective of image semantic segmentation. The major difference between the semantic segmentation method based on a convolutional neural network and the traditional semantic segmentation method is that the network can automatically learn the image features and carry out end-to-end classification learning, which greatly improves the accuracy and efficiency of image semantic segmentation.

U-Net [16] network (see Figure 3(a)) has good performance in medical image segmentation and is superior to other coding-decoding structure networks in small target segmentation performance. Therefore, the U-Net network is selected as the main model to segment the fissured tongue images in traditional Chinese medicine. Due to the influence of light intensity, diet, and drugs, the tongue image is characterized by a large amount of information and many features. FCN [7] and SegNet [18] networks are not fine enough for crack segmentation in traditional Chinese medicine tongue image, and it is easy to lose detailed information. Compared with them, the U-Net network can obtain a better segmentation effect. Therefore, this study proposes improving the U-Net network structure to solve the problem that small targets are difficult to be accurately segmented.

Compared with U-Net, the improved U-Net model uses pretrained GoogLeNet as the feature extraction network for image feature extraction. After feature extraction, feature information is added through the GCN module and BR module. Through this operation, the decoder can recover the image details and spatial dimension better by an upsampling operation. The improved U-Net network increases the size of the receptive domain by effectively increasing the size of the convolution kernel and improves the segmentation accuracy of small targets.

The improved U-Net model still retains the encoder-decoder structure, as shown in Figure 3(c). The improved U-Net model encoder adopts GoogLeNet as the pretraining network. The left half of Figure 3(c) is the encoder part composed of the GoogLeNet network. This part is mainly composed of four submodules. The submodule contains the Inception module, which extracts the features of the input image through pooling operation. The final output of the GoogLeNet encoder enters the GCN module. Then, while the output of the GCN module is upsampled, the channel number is added to the output of its previous submodule. The output result enters the BR module as the input of the next upsampling, and so on. Finally, the model outputs the semantic segmentation prediction graph.

On balance, according to Chao's analysis on classification and segmentation in images, we have known that large kernels are vital to relieving the contradiction between classification and localization. Following the principle of large-size kernels, we add the Global Convolutional Network (GCN) module in the U-Net structure. In addition, to further refine the object boundaries, we also add a Boundary Refinement (BR) block. Qualitatively, the GCN module mainly optimizes the internal structure of the network while the BR block increases performance near boundaries which can precisely capture the edge information of the image. The experiments in Section 4 show that our proposed improved U-Net structure achieves good performance, which realizes the fissure extraction and meets a good trade-off between valid receptive filed and the number of parameters.

## 4. Experimental Evaluation and Discussion

### 4.1. Datasets

At present, there is no fully public dataset of tongue images. Therefore, a new dataset is proposed as a reference for fissured tongue images segmentation in this study. The fissured tongue was judged by strictly referring to the 12th Five-Year Plan textbooks for the higher education of Chinese medicine industry in China, such as The Tongue Image Discrimination of Traditional Chinese Medicine [15] and the tongue Diagnosis Chapter of Diagnostics of Traditional Chinese Medicine [34]. The images were also evaluated and confirmed by TCM physicians for consistency. In this study, a total of 316 clinical tongue images conforming to fissured tongue images were collected and screened in JPG format. Unified coding was carried out for the selected tongue image data. Meanwhile, Photoshop CC 2019 was used to quickly further crop the selected tongue images and retain the regions containing the tongue images for preprocessing. After cutting, the tongue image is shown in Figure 4.

Labelme_3.16.7 image annotation software based on Python was used to annotate the crack area of the tongue image. Each tongue image generates the corresponding annotated JSON file and then transforms the JSON file through the program to generate the corresponding semantic label image of the tongue image. In order to ensure the accuracy of data annotation, we also check and confirm the annotation. All the annotated data were randomly divided into training verification set and test set according to the ratio of 7 : 3, in which there were 223 training verification datasets and 93 test datasets. During the experiment, in order to avoid the overfitting problem, we amplified the data of the training verification data set through the geometric transformation of the image, including the data enhancement operations such as flipping transformation and random pruning. We balanced the number of sampled images and randomly divided them into training sets and verification sets according to the ratio of 7 : 3, among which there were 1413 training sets and 596 training sets. The data preprocessing results during the experiment are shown in Figure 4.

The experimental system including the pretraining network is based on the Pytorch framework, and all the experiments are completed on NVIDIA-GP 1060 (6G) graphics card, CUDA_verision 10.1, and Python version 3.6. During the training time, we train Adam with momentum. We use a minibatch size of 4 images and fixed initial learning rates of 1 × 10^−5^. We use momentum 0.9, and the learning rate is set to gradually decrease with the increase of epoch to achieve a better training effect. We set the size of the input image to 256 × 256. The performance is measured by standard mean intersection over union (MIoU) [35].

### 4.2. Comparison with Different Classification Models without Pretraining

U-Net Network model is mainly composed of Encoder Network and Decoder Network. The encoder network converts the high-dimensional vector into the low-dimensional vector to realize the low-dimensional extraction of high-dimensional features. The encoder network captures more translation-invariant features through multiple maximum pooling operations, but it also loses more important segmentation bases such as the boundary information of the feature map. Therefore, different pretraining networks are used for feature extraction in the encoder part of the U-Net model, and the algorithm accuracy of the model in the process of training and verification is compared, as well as the segmentation effect in the test process. During the experiment, the hyperparameter settings of the network, such as the learning rate, are guaranteed to be the same. The comparative experimental results are shown in Figure 5, and the segmentation prediction results are shown in Figure 6. As can be seen from the prediction results of different pretraining networks, compared with ResNet, VGGNet, DenseNet [36], ShuffleNet [37], and SEResNet networks, the GoogLeNet network is more suitable for U-Net encoder in this study and has a better segmentation effect.

### 4.3. Model Comparison with or without GCN Module

In Section 2.3, we demonstrate that the GCN module improves the classification capability of the segmentation model by introducing dense connections into the feature map to help cope with a large number of transformations. To further prove this point, we carry out experiments to verify the effectiveness of integrating the GCN module and BR module in the network. In this study, we add fusion GCN module and BR module to VGGNet_Unet, GoogLeNet_Unet, and SEResNet_Unet, respectively. Before feature fusion, the output results of each feature extraction submodule of the encoder are first put into the GCN module and then added with the upsampling results of the decoder. Finally, the added results are put into a BR module, and so on. The experimental comparison was conducted in the test dataset, and the experimental results are shown in Table 1. As can be seen from Table 1, compared with the model without GCN and BR modules, the tongue image crack segmentation accuracy of the model with GCN and BR modules is improved, and the MIoU of the GoogLeNet_Unet model with GCN and BR modules in tongue image crack segmentation is increased by 5.3%. This shows that the GCN module and BR module applied to the semantic segmentation of tongue image crack can better fuse the multiscale image context information, to effectively utilize the feature information of the image and obtain higher accuracy of network prediction.

### 4.4. Comparison of Different Convolutions in GCN Module

In this section, we mainly discuss the experiments using deep separable convolution instead of ordinary convolution in the GCN module (labeled GCN_D). Since Sifre et al. [38] proposed in 2013 that interchannel and spatial correlations of the convolutional layer are recoupable coupled, deeply separable convolution has been a key building block for many efficient neural network frameworks to achieve model lightweight. The difference between ordinary convolution and deeply separable convolution mainly lies in that ordinary convolution considers all channels in the corresponding region at the same time, deep separable convolution uses different convolutions to check different channels for convolution, and ordinary convolution is divided into two independent parallel convolution processes, Depthwise [39] convolution and Pointwise [39] convolution. Based on the previous chapter, we adopt the same experimental environment and add the GCN_D module and BR module, respectively, for VGGNet_Unet, GoogLeNet_Unet, and SEResNet_Unet. The experimental comparison was conducted in the same test dataset, and the experimental results are shown in Table 2. As can be seen from Table 2, the tongue image crack segmentation accuracy of the model with the GCN_D module is not significantly different from that of the model with the GCN module. This indicates that whether deep separable convolution is used for semantic segmentation of tongue image crack in the GCN module has little influence.

### 4.5. Experimental Results on Test Datasets

In this study, we conducted experiments on some outstanding models, such as FCN, DeepLab v3_plus [23], FRN [24], SegNet [18], and so on [40–42], VGGNet_Unet, and the improved U-Net in the test dataset with the weights obtained in the training process. The experimental results are shown in Figure 7, and the prediction results are shown in Figure 8. It can be seen that neither Deeplab3_plus nor FCN model can extract tongue image cracks well, especially in the case of small and not obvious crack features in tongue image; the prediction effect is poor and even cannot predict accurately. GoogLeNet_Unet and the improved U-Net can better distinguish the tongue image cracks from the background in the area where the tongue image cracks are sparse. Compared with the classical U-Net model, the improved U-Net network not only reduces the error rate but also improves the predicted MIoU. To better display the experimental results, we randomly selected three pieces of data from the dataset, used the improved U-Net network to predict these pictures through the weight obtained in the training process, and superimposed the prediction results on the original image to better illustrate the segmentation effect of the network, as shown in Figure 9.

### 4.6. Model Validation

In this section, an experiment was described to validate the improved model and other models. The overall flow of the experiment is shown in Figure 10. The first step is to collect tongue images. Generally, tongue images need to be taken by mobile phones, digital cameras, and other pieces of equipment in a closed, stable, and fixed acquisition environment. Secondly, we will give the collected tongue images to professional doctors for identification to judge whether the collected image data can be used in the experiment. Because the collected tongue images usually contain redundant backgrounds such as teeth, lips, and face, it has a great impact on the later experimental analysis. We need to remove the interference background from the collected tongue image to segment the analyzable tongue image. This is the most critical step in the experiment. Finally, we send the processed tongue image into the pretrained model in Section 4.5 for feature extraction of fissured tongue images.

In this experiment, the crack tongue image we selected is neither in the training dataset nor in the test dataset, which ensures the effectiveness of the verification experiment. In Figure 11, we show the prediction results of a fissured tongue picture. The experimental results show that FCN, DenseNet_Unet, VGGNet_Unet, GoogLeNet_Unet, and the improved U-Net model can accurately extract crack features.

## 5. Conclusions

Tongue crack is an important feature of tongue states. Not only does change of tongue crack states reflect objectively and accurately changed circumstances of some typical diseases and TCM syndrome but also semantic segmentation of the fissured tongue can combine the other features of tongue states to further improve tongue diagnosis systems identification accuracy. Although computer tongue diagnosis technology has made great progress, there are few studies on the fissured tongue, and most of them focus on the analysis of tongue coating and body. Moreover, research fruits of semantic segmentation of fissured tongue would accelerate practical research on tongue crack in computerized tongue diagnosis and also possess potential application in medical clinic practice simultaneously.

Furthermore, deep learning has had a tremendous impact on various fields in science [43]. The focus of the current study is on one of the most critical areas of computer vision: medical computer vision, particularly deep learning-based approaches for medical image segmentation. In the field of medical image segmentation, deep correlation technology has been mature and has broad application prospects. It has been applied to lung image segmentation [44], brain tumor and other tissues segmentation [45], cell and membrane structure segmentation [46, 47], bone tissue segmentation [48], and tibia cartilage segmentation [49]. At present, some frameworks for specific segmentation tasks have been formed, and good results have been obtained, but further optimization is needed to improve the segmentation accuracy. Therefore, compared with the traditional image recognition method, deep learning technology can more accurately complete fissured tongue segmentation and be conducive to the automatic recognition of TCM tongue images.

In this study, we propose an image semantic segmentation model based on the U-Net model to detect fissured tongue images and compare the different pretraining networks for the encoder part and whether to add the GCN module and BR module. The improved U-Net model achieves 47.5% semantic segmentation accuracy of fissured tongue images, which is 15.1% higher than the FCN model, 30.5% higher than the SegNet model, 5.3% higher than the VGGNet_Unet model, and 1.8% higher than GoogLeNet_Unet model. At the same time, the improved U-Net model can capture the multiscale context information of the image under the multisampling rate, with high computational efficiency, and it can effectively complete the crack detection on the tongue image dataset. Although the improved U-Net model has been greatly improved to a certain extent, the experiment also has some limitations. It can be seen from the performance of the model on the test dataset that the model still needs to be improved. At the same time, the mapping from input to output in the learning process of a neural network is discontinuous [50]. This discontinuity makes the picture can deceive the model and produce wrong judgment after appropriate modification [51]. In the follow-up work, we need to conduct adversarial example attack experiments on the model and modify the training samples [52]. By adding more adversarial samples to the training set, we can effectively avoid some attacks. We can test the model by adding a small amount of noise that cannot be detected by human eyes on the basis of clean data. In the encoder design part, we can add additional networks on the basis of the GoogLeNet network to keep the original network unchanged.

In the future, the research on computerized fissured tongue diagnosis can be further improved and studied from the following aspects. (1) Feature extraction: defining and extracting more crack features is the top priority of computerized fissured tongue diagnosis in the future. In the future computer tongue diagnosis system, TCM tongue diagnosis can be assisted by using only the mapping relationship between the shape characteristics of tongue cracks and clinical diseases, which further simplifies the steps of computer tongue crack diagnosis. (2) Feature fusion: computer tongue diagnosis and computerized tongue crack diagnosis are combined with other diagnostic methods to promote the objective research of four diagnoses in traditional Chinese medicine. (3) System integration and testing: integrating the research results of computer fissured tongue diagnosis into the system and conducting large-scale clinical tests in some hospitals is a key step for computer tongue diagnosis technology to go to the market. Among them, the “AI Open Platform for Traditional Chinese Medicine Tongue Diagnosis” jointly developed by Anhui University of Chinese medicine and a company in Hefei is a typical case. The system integrates tongue image acquisition, tongue image diagnosis, operation interface, and system advantages. Compared with other traditional tongue diagnosis instruments, it is a relatively complete computer-aided tongue diagnosis system. Moreover, the application of computer tongue diagnostics to mobile is also the mainstream trend. In this process [53], we analyze the concepts of security, privacy, and resilience, along with their relationships in detail, and formulate a set of principles for designing a mobile application linking resilience and security in privacy protection.

## Figures and Tables

**Figure 1:** Inception module with dimensionality reduction from the GoogLeNet architecture.

**Figure 2:** Residual block from the ResNet architecture.

**Figure 3:** The 3D U-Net architecture. Blue boxes represent feature maps. The number of channels is denoted above each feature map. (a) U-Net network structure, (b) GCR module and BR module, and (c) improved U-Net network structure.

**Figure 4:** Six cases of fissured tongue images and data preprocessing results: (a) the cracks in the picture are evenly distributed and obvious; (b) the cracks in the picture are scattered and obvious; (c, d) the crack distribution in the picture is scattered and not obvious; (e) the cracks in the picture are widely distributed and obvious, which is difficult to segment; (f) the crack distribution in the picture is single and easy to segment.

**Figure 5:** A different pretraining net comparison.

**Figure 6:** Different pretraining as encoder part of prediction result.

**Figure 7:** Comparison of MIoU between classical segmentation model and improved U-Net model in the test dataset.

**Figure 8:** Segmentation prediction results of different models in the test dataset.

**Figure 9:** Overlay effect of the original picture and predicted segmentation result image.

**Figure 10:** Experimental flow chart of validation model.

**Figure 11:** The experimental prediction results of six models with high MIoU in Section 4.5.

**Table 1:** Model comparison with or without the GCN module and BR module.

Model	PA (pixel accuracy)	Loss (%)	MIoU (mean intersection over union)
SEResNet_Unet	98.5	4.96	38.0
SEResNet_GCN_Unet	98.5	5.10	43.1
VGGNet_Unet	98.6	4.32	42.0
VGGNet_GCN_Unet	98.6	4.84	46.2
GoogLeNet_Unet	98.6	4.11	45.5
GoogLeNet_GCN_Unet	98.7	4.48	47.3

**Table 2:** Model comparison of different convolutions in GCN module.

Model	PA (pixel accuracy)	Loss (%)	MIoU (mean intersection over union)
SEResNet_GCN_Unet	98.5	5.10	43.1
SEResNet_GCND_Unet	98.5	5.19	39.6
VGGNet_GCN_Unet	98.6	4.84	46.2
VGGNet_GCND_Unet	98.6	4.46	46.2
GoogLeNet_GCN_Unet	98.7	4.48	47.3
GoogLeNet_GCND_Unet	98.6	4.02	47.5

## Data Availability

The data presented in this study are available on request from the corresponding author.
